The article "Factors Affecting the Readmission of Patients with Pancreatic Cancer after Surgery" was retracted in 2023. Reasons: signs of a paper mill; compromised peer review; unreliable results or conclusions.

# Factors Affecting the Readmission of Patients with Pancreatic Cancer after Surgery

**DOI:** 10.1155/2022/6106914

**Published:** 2022-04-29

**Authors:** Xiaojing Gu, Wei Zhou, Juan Han

**Affiliations:** ^1^Department of Biliary and Pancreatic Surgery, Tongji Hospital Affiliated to Tongji Medical College, Huazhong University of Science and Technology, Wuhan, Hubei 430030, China; ^2^Wuhan Polytechnic University, Wuhan, Hubei 430023, China

## Abstract

**Objective:**

Pancreatic cancer is one of the deadliest solid malignancies. Its surgical resection is technically very challenging and has a high risk of complications even after discharge. This study analyzed the risk factors associated with unplanned readmission after pancreatic cancer surgery.

**Methods:**

Pancreatic cancer patients who were readmitted within 30 days after surgery were classified as the observation group, while those not readmitted within 30 days postsurgery were classified as the control group. The serum levels of gastrointestinal hormones, stress hormones, and peripheral immune cells of the two groups were compared at different intervals.

**Results:**

No significant differences in gender and age were observed between the two groups. At 7, 14, and 21 days postsurgery, the levels of gastrointestinal hormones motilin, gastrin, calcitonin gene-related peptide, and growth hormone-releasing peptide of the observation group were lower than the control group, while the levels of adrenocorticotropin, renin, angiotensin, and plasma aldosterone of the observation group were significantly higher than the control group. In addition, compared to the control group, lower levels of CD4+T cells, CD8+T cells, and NKT cells and higher levels of Treg, Breg, and MDSC cells were observed in the peripheral blood of the observation group.

**Conclusion:**

The serum levels of gastrointestinal hormones, stress hormones, and peripheral immune cells could be associated with the risk of unplanned readmission within 30 days after pancreatic cancer surgery.

## 1. Introduction

Pancreatic cancer is one of the deadliest human cancers [1] and has a very poor 5-year survival rate [2]. Studies have shown that smoking, alcohol consumption, dietary factors, diabetes, obesity, and genetics are important factors associated with the incidence of pancreatic cancer [3, 4]. At present, surgical resection followed by adjuvant systemic chemotherapy represents the only chance for long-term survival [5]. However, the surgical resection of pancreatic cancer may induce or exacerbate nutritional and metabolic dysfunction in patients, which may adversely affect their quality of life [6].

Previous studies have shown that postoperative nutritional imbalance was associated with the postoperative death of approximately 10% of pancreatic cancer patients [7, 8]. Further, inadequate nutritional intake was found to be associated with increased stress response, slow wound healing, and high postoperative infection rates, which could lead to higher risks for readmission [9, 10]. Thus, we hypothesized that the readmission of pancreatic cancer patients after surgery could be associated with gastrointestinal factors, stress responses, and immune status.

The article "Factors Affecting the Readmission of Patients with Pancreatic Cancer after Surgery" was retracted in 2023. Reasons: signs of a paper mill; compromised peer review; unreliable results or conclusions.

Recently, unexpected readmissions after surgery have become a focus of attention for measuring the quality of care [11]. Readmission within 30 days of surgery puts additional strain on the healthcare systems and has been shown to negatively affect patient's quality of life. Kent et al. [12] found that a single readmission after pancreatic resection could cost an average of $16,000 or more, and in addition to the financial impact of readmission, the unplanned readmission of patients to the hospital further limited hospital resources. Most readmissions after surgery are due to medical conditions [13]. In a study by Kassin et al. [14], the authors found that the risk factors for readmission after general surgery were primarily due to the occurrence of complications. Therefore, identifying factors closely associated with the greatest risk for postoperative readmission could help clinicians carefully assess these parameters before and after surgery to reduce the risk of readmissions and improve patients' prognoses.

Currently, research on the causes of unplanned postoperative readmissions in patients with pancreatic cancer is limited. In this study, we examined the factors associated with 30-day postoperative readmission in pancreatic cancer patients who underwent pancreatic surgery.

## 2. Materials and Methods

### 2.1. Study Population

The data of patients who were diagnosed with pancreatic cancer and underwent pancreatic cancer surgery at the Tongji Hospital Affiliated to Tongji Medical College, Huazhong University of Science and Technology (Wuhan, China) from February 2019 to March 2020 were retrieved. Patients were selected based on the following inclusion criteria: ① The diagnosis of pancreatic cancer was made based on the guidelines for diagnosis and treatment of pancreatic cancer published by the Ministry of Health in 2011 [15]; ② the patients had no mental abnormality and could independently take care of themselves; ③ provided informed consent; and ④ had a postoperative survival time of more than 3 months. Cases were excluded if they ① had severe cardiopulmonary insufficiency; ② hepatorenal dysfunction; ③ hyperthyroidism; ④ cardiopulmonary insufficiency; or ⑤ pregnancy. Patients who were readmitted within 30 days after surgery were classified into the observation group, and those who were not readmitted within 30 days after surgery were classified into the control group. This study was approved by the Ethics Committee of Tongji Hospital Affiliated to Tongji Medical College, Huazhong University of Science and Technology (TJ-IRB20190418).

The article "Factors Affecting the Readmission of Patients with Pancreatic Cancer after Surgery" was retracted in 2023. Reasons: signs of a paper mill; compromised peer review; unreliable results or conclusions.

### 2.2. Detection Method

To assess the gastrointestinal function, stress response, and immune status of the patients, their corresponding serum hormones levels, i.e., motilin (MTL), gastrin (GAS), calcitonin gene-related peptide (CGRP), growth hormone-releasing peptide (Ghrelin), adrenocorticotropin (ACTH), renin (R), angiotensin (AT-II) and plasma aldosterone (ALD), cluster of differentiation (CD) 4+T cells, CD8+T cells, natural killer T cell (NKT), regulatory T cell (Treg), regulatory B cell (Breg), and myeloid-derived suppressor cell (MDSC), were investigated. The gastrointestinal function and stress response-related hormones levels were measured using enzyme-linked immunosorbent assay (ELISA). The immune cells were detected by Beckman Coulter CytoFLEX flow cytometry. All hormones were measured before surgery, and 7, 14, and 21 days after surgery. Briefly, 3 mL of the patients' peripheral venous blood was collected at the indicated time and the gastrointestinal, stress response, and immune related parameters were measured using ELISA or Beckman Coulter CytoFLEX flow cytometry.

### 2.3. Statistical Analysis

The Statistical Package for the Social Sciences (SPSS, version 22.0; IBM, New York, United States) software was used for statistical analysis. Categorical variables were expressed as frequency and percentage (%), and the comparison between groups was expressed by the *χ*^2^ test. The measurement data were expressed as mean ± standard deviation (SD), and the comparison between groups was performed using the independent sample *t*-test. *P* < 0.05 indicated that the difference between comparisons was statistically significant.

## 3. Results

### 3.1. Patients' Information

A total of 87 (observation group [*n* = 41] and control group [*n* = 46]) pancreatic cancer patients were eligible for this study. In the observation group, there were 23 males and 18 females. They were from 44 to 69 years old and had an average age of 57.06 ± 10.25 years. In the control group, there were 24 males and 22 females. They were from 45 to 70 years old and had an average age of 57.74 ± 10.64 years. There was no significant difference in the general data between the two groups (*P* > 0.05).

### 3.2. Comparison of Gastrointestinal Hormones at Different Time Intervals

The hormones MTL, GAS, CGRP, and Ghrelin secreted by the gastrointestinal tract were measured to reflect the gastrointestinal function. As shown in Table 1, there was no significant difference in serum gastrointestinal hormone levels between the two groups before surgery. However, the levels of MTL, GAS, CGRP, and Ghrelin in the observation group were significantly lower than the control group at 7, 14, and 21 days after surgery (*P* < 0.05).

The article "Factors Affecting the Readmission of Patients with Pancreatic Cancer after Surgery" was retracted in 2023. Reasons: signs of a paper mill; compromised peer review; unreliable results or conclusions.

### 3.3. Comparison of Stress Hormones at Different Time Intervals

In this study, the hormones, ACTH, R, AT-II, and ALD, associated with stress response were measured. Our results showed that there was no significant difference in serum stress hormone levels between the two groups before surgery, but the levels of ACTH, R, AT-II, and ALD in the observation group were significantly higher than the control group at 7, 14, and 21 days after surgery (*P* < 0.05; Table 2).

### 3.4. Comparison of Immune Cells in the Peripheral Blood at Different Time Intervals

Here, the levels of CD4+T cells, CD8+T cells, NKT cells, Treg, Breg, and MDSC were measured to reflect the patients' autoimmune status. As shown in Tables 3 and 4, the levels of these immune cells between the two groups were well-balanced before surgery. However, at 7, 14, and 21 days after surgery, the levels of CD4+T cells, CD8+T cells, and NKT cells in the observation group were found to be lower than those in the control group (Table 3), while the levels of Treg, Breg, and MDSC cells in the observation group were higher than the control group (Table 4).

## 4. Discussion

In this study, we found that the serum levels of gastrointestinal hormones, stress hormones, and immune cells between the observation and control group were well-balanced before surgery but changed significantly at different postoperative time intervals.

Studies have shown that anomalies in the secretion of gastrointestinal hormones after cancer surgery are important factors that affect changes in gastrointestinal functions [16]. The gastrointestinal hormones MTL and Ghrelin are secreted by the intestine during the fasting phase and can promote complex gastrointestinal motility [17–19]. Gastrin can indirectly promote hydrochloric acid secretion from gastric cells and accelerates gastrointestinal motility [20]. CGRP can regulate gastric mucosal vascular and smooth muscle contraction and affects gastric acid secretion [21]. In this present study, we found that the serum levels of MTL, GAS, CGRP, and Ghrelin were significantly lower in the pancreatic cancer patients who were readmitted within 30 days after surgery than those in the control group at 7, 14, and 21 days after surgery. Upon investigating the nutritional status of 105 postoperative patients with pancreatic cancer, Zhang et al. [22] found that compared with other general surgery malignancies, pancreatic cancer patients had a higher incidence of malnutrition, suggesting malnutrition as an understudied complication of pancreatic cancer. In a study by Elliott et al. [23], the mean fasting Ghrelin levels in patients with esophageal cancer were found to decline from day 10 till one year after surgery. La Torre et al. [24] conducted a nutritional risk assessment for patients undergoing pancreatic cancer surgery and found that postoperative complication rate, mortality, and infection rate were significantly increased in patients with poor nutrition levels. These studies indicate that gastrointestinal hormone secretion is an important factor affecting postoperative readmission of pancreatic cancer.

The article "Factors Affecting the Readmission of Patients with Pancreatic Cancer after Surgery" was retracted in 2023. Reasons: signs of a paper mill; compromised peer review; unreliable results or conclusions.

The surgical procedure for pancreatic cancer is technically challenging and is associated with significant trauma. In addition, the postoperative period is prone to stress and hormonal disorders, and these patients require intensive postoperative care due to the high risks of complications [25]. Stress activates the hypothalamic-pituitary-adrenal axis and the sympathetic-adrenal medulla, leading to the secretion of ACTH, which affects the adrenal cortex and promotes the synthesis and secretion of corticotropin-releasing hormone [26]. The renin-angiotensin-aldosterone system (RAAS) can regulate vasoconstriction during stress response, and the initial link of the system is an increase in R secretion, which acts on AT-I to form AT-II [27]. AT-II can accelerate vasoconstriction and can also increase the secretion of ALD [28]. Studies have demonstrated that stress hormones are associated with postoperative infections and delayed postoperative recovery [29]. In this study, the levels of ACTH, R, AT-II, and ALD in the observation group were found to be significantly higher than those in the control group at 7, 14, and 21 days after surgery. Chi et al. [30] reported that postoperative tea therapy in elderly patients could significantly reduce the serum levels of ACTH and COR, thereby, reducing perioperative stress and promoting postoperative recovery. These studies suggest that the aggravation of stress reaction and impairment of immune function caused by malnutrition were the predictive factors of postoperative readmission for pancreatic cancer.

Further, in this study, on the 7th, 14th, and 21st day after surgery, the levels of CD4+T cells, CD8+T cells, and NKT cells in the peripheral blood of the observation group were lower than those of the control group, while higher levels of Treg, Breg, and MDSC cells were observed in the observation group. Studies have shown that surgery is an invasive procedure associated with acute inflammation and immune responses that can increase the risk of postoperative complications [31]. Ding et al. [32] found that preoperative nutritional support could improve the nutritional status and immune function of patients with gastric cancer after surgery, alleviate the inflammatory response, and promote patient recovery. In a clinical study by Zhou et al. [33], the authors found that patients with good prognosis after aneurysmal subarachnoid hemorrhage had significantly higher proportions of CD4+T cells, CD8+T cells, and NKT than those with poor prognosis. These studies suggest that postoperative suppression of immune function could therefore affect the clinical prognosis of postoperative patients. Thus, based on the above findings and current literature, to reduce the risk of malnutrition and readmission, we suggest that the serum levels of gastrointestinal hormones, stress hormones, and immune cells should be investigated before and after surgery and adequately compensated based on the patient's requirements.

The article "Factors Affecting the Readmission of Patients with Pancreatic Cancer after Surgery" was retracted in 2023. Reasons: signs of a paper mill; compromised peer review; unreliable results or conclusions.

In conclusion, this study findings showed that the serum levels of gastrointestinal hormones, stress hormones, and peripheral blood immune cells could be relevant factors associated with unplanned readmission within 30 days after pancreatic cancer surgery. To reduce the risk of readmission, personalized clinical nutrition interventions before and after surgery could be implemented to timely counteract malnutrition in these patients. To validate these findings, further investigations using a larger cohort of patients in prospective settings are required.

## Figures and Tables

**Table 1:** Comparison of gastrointestinal hormone contents at different postoperative intervals (pg/mL).

Group	Time	MTL	GAS	CGRP	Ghrelin
Observation group (*n* = 41)	Before operation	238.13 ± 36.16	185.21 ± 21.36	108.26 ± 13.27	74.68 ± 9.72
	7 days after operation	139.55 ± 15.63^∗^^#^	93.54 ± 11.57^∗^^#^	60.32 ± 8.551^∗^^#^	33.46 ± 5.25^∗^^#^
	14 days after operation	147.39 ± 17.83^∗^^#^	107.51 ± 14.29^∗^^#^	64.39 ± 9.52^∗^^#^	45.21 ± 6.74^∗^^#^
	21 days after operation	163.87 ± 19.31^∗^^#^	112.49 ± 14.28^∗^^#^	69.17 ± 9.64^∗^^#^	48.32 ± 6.81^∗^^#^
Control group (*n* = 46)	Before operation	235.41 ± 33.27	183.47 ± 22.15	107.45 ± 14.52	75.22 ± 9.36
	7 days after operation	173.52 ± 20.35^∗^	132.36 ± 17.83^∗^	75.42 ± 9.35^∗^	46.54 ± 7.25^∗^
	14 days after operation	196.18 ± 26.39^∗^	141.39 ± 16.58^∗^	79.39 ± 9.87^∗^	54.39 ± 7.56^∗^
	21 days after operation	205.46 ± 28.39^∗^	149.52 ± 17.28^∗^	83.39 ± 11.17^∗^	59.82 ± 7.64^∗^

Values are presented as mean ± SD. ^∗^*P* < 0.05 vs. before operation; ^#^*P* < 0.05 vs. control group. MTL: Motilin; GAS: Gastrin; CGRP: Calcitonin gene-related peptide; Ghrelin: Growth hormone-releasing peptide.

The article "Factors Affecting the Readmission of Patients with Pancreatic Cancer after Surgery" was retracted in 2023. Reasons: signs of a paper mill; compromised peer review; unreliable results or conclusions.

**Table 2:** Comparison of stress hormone contents at different postoperative intervals.

Group	Time	ACTH (pmol/L)	R (ng/mL)	AT-II (pg/mL)	ALD (pg/mL)
Observation group (*n* = 41)	Before operation	3.04 ± 0.43	1.94 ± 0.23	2.92 ± 0.49	255.32 ± 31.31
	7 days after operation	6.26 ± 0.84^∗^^#^	4.32 ± 0.58^∗^^#^	5.58 ± 0.82^∗^^#^	486.62 ± 62.36^∗^^#^
	14 days after operation	5.96 ± 0.81^∗^^#^	4.01 ± 0.52^∗^^#^	5.03 ± 0.61^∗^^#^	451.37 ± 59.02^∗^^#^
	21 days after operation	5.43 ± 0.78^∗^^#^	3.86 ± 0.45^∗^^#^	4.85 ± 0.58^∗^^#^	423.43 ± 55.63^∗^^#^
Control group (*n* = 46)	Before operation	2.93 ± 0.42	1.88 ± 0.26	2.86 ± 0.55	256.52 ± 33.53
	7 days after operation	4.62 ± 0.75^∗^	3.28 ± 0.45^∗^	4.28 ± 0.55^∗^	378.81 ± 41.24^∗^
	14 days after operation	4.32 ± 0.54^∗^	3.03 ± 0.39^∗^	4.02 ± 0.53^∗^	341.29 ± 39.27^∗^
	21 days after operation	4.15 ± 0.55^∗^	2.75 ± 0.36^∗^	3.72 ± 0.51^∗^	313.53 ± 36.79^∗^

Values are presented as mean ± SD. ^∗^*P* < 0.05 vs. before operation; ^#^*P* < 0.05 vs. control group. ACTH: Adrenocorticotropin; R: Renin; AT-II: Angiotensin; ALD: Aldosterone.

**Table 3:** Comparison of the content of immune cells in peripheral blood at different postoperative intervals.

Group	Time	CD4+T cells	CD8+T cells	NKT cells
Observation group(*n* = 41)	Before operation	43.78 ± 6.04	38.02 ± 5.62	1.22 ± 0.18
	7 days after operation	30.22 ± 3.59^∗^^#^	27.55 ± 3.26^∗^^#^	0.79 ± 0.08^∗^^#^
	14 days after operation	31.27 ± 4.49^∗^^#^	29.01 ± 3.47^∗^^#^	0.86 ± 0.11^∗^^#^
	21 days after operation	33.54 ± 4.49^∗^^#^	31.22 ± 3.59^∗^^#^	0.91 ± 0.19^∗^^#^
Control group (*n* = 46)	Before operation	43.16 ± 5.96	37.58 ± 5.29	1.19 ± 0.18
	7 days after operation	35.62 ± 4.48^∗^	31.04 ± 4.59^∗^	0.82 ± 0.13^∗^
	14 days after operation	37.42 ± 5.53^∗^	33.55 ± 5.08^∗^	1.05 ± 0.16^∗^
	21 days after operation	39.73 ± 6.17^∗^	35.27 ± 5.64^∗^	1.13 ± 0.17^∗^

Values are presented as mean ± SD. ^∗^*P* < 0.05 vs. before operation; ^#^*P* < 0.05 vs. control group.

**Table 4:** Comparison of the content of immune cells in peripheral blood in different periods.

Group	Time	Treg	Breg	MDSC
Observation group(*n* = 41)	Before operation	3.46 ± 0.49	4.32 ± 0.58	2.09 ± 0.33
	7 days after operation	7.05 ± 0.89^∗^^#^	8.51 ± 1.03^∗^^#^	4.48 ± 0.59^∗^^#^
	14 days after operation	6.67 ± 0.81^∗^^#^	7.62 ± 0.89^∗^^#^	3.83 ± 0.45^∗^^#^
	21 days after operation	5.93 ± 0.75^∗^^#^	7.01 ± 0.71^∗^^#^	3.42 ± 0.41^∗^^#^
Control group (*n* = 46)	Before operation	3.42 ± 0.46	4.29 ± 0.53	2.04 ± 0.36
	7 days after operation	4.99 ± 0.75^∗^	6.89 ± 0.78^∗^	3.27 ± 0.53^∗^
	14 days after operation	4.51 ± 0.63^∗^	6.04 ± 0.67^∗^	3.04 ± 0.46^∗^
	21 days after operation	4.13 ± 0.48^∗^	5.42 ± 0.68^∗^	2.78 ± 0.38^∗^

Values are presented as mean ± SD. ^∗^*P* < 0.05 vs. before operation; ^#^*P* < 0.05 vs. control group. Treg: Regulatory T cell; Breg: Regulatory B cell; MDSC: Myeloid-derived suppressor cell.

The article "Factors Affecting the Readmission of Patients with Pancreatic Cancer after Surgery" was retracted in 2023. Reasons: signs of a paper mill; compromised peer review; unreliable results or conclusions.

## Data Availability

The data used to support the findings of this study are available from the corresponding author upon request.
